The article "Analysis on the Effect of Different Surgical Methods on the Treatment of Senile Osteoporotic Spinal Compression Fractures and the Influencing Factors of Complications" was retracted in 2023. Reasons: unreliable results or conclusions; concerns about the data; concerns about the peer review; concerns about the citations.

# Analysis on the Effect of Different Surgical Methods on the Treatment of Senile Osteoporotic Spinal Compression Fractures and the Influencing Factors of Complications

**DOI:** 10.1155/2021/1599470

**Published:** 2021-08-31

**Authors:** Dejun Yu, Zuyao Liu, Hongqing Wang, Ran Yao, Fu Li, Yang Yang, Fenglong Sun

**Affiliations:** ^1^Department of Orthopaedics, Beijing Rehabilitation Hospital, Capital University of Medical Sciences, Beijing 100144, China; ^2^Department of Orthopaedic Rehabilitation Center, Beijing Rehabilitation Hospital, Capital University of Medical Sciences, Beijing 100144, China

## Abstract

Osteoporotic fractures are a common type of fractures in the elderly, among which spinal compression fractures are more common. After the occurrence of fractures, due to the compression and burst of the vertebral body, this will lead to local kyphosis deformity and even affect the balance of the sagittal spine. In the past, conservative treatments were used for osteoporotic spinal compression fractures. Although it can relieve pain symptoms, it can easily lead to complications such as aggravation of osteoporosis and deep vein thrombosis of the lower extremities. At present, percutaneous vertebroplasty (PVP) and percutaneous kyphoplasty (PKP) are the main clinical surgical treatments, both of which are minimally invasive surgery, short operation time, effective pain relief, and rapid postoperative recovery. Although both of them are effective, there is still controversy over the efficacy of both in the treatment of osteoporotic spinal compression fractures. The purpose of this study was to investigate the efficacy of PVP and PKP in the treatment of elderly osteoporotic spinal compression fractures and to analyze the related factors that affect the occurrence of postoperative complications. The results show that both PVP and PKP can effectively improve the pain and dysfunction of elderly patients with osteoporotic spinal compression fracture, restoration of vertebral height, and correct kyphosis, but PKP has better effect and higher safety and is worth promoting. Postoperative complications of patients are related to their age, bone mineral density, use of hormones, and antiosteoporosis treatment.

## 1. Introduction

Osteoporosis is a systemic skeletal system disease that causes bone fractures in various parts of the body due to the destruction of bone microstructure and low bone mass, which leads to increased bone fragility [1, 2]. Osteoporotic fracture is a type of fracture commonly found in the elderly population, among which spinal compression fracture is more common. After fracture occurs, the compression and burst of the vertebral body will lead to local kyphosis, even affecting the balance of the sagittal plane of the spine [3–6]. At present, the clinical use of surgical treatment, percutaneous vertebroplasty (PVP), is one of its routine surgery, the operation through the image guided percutaneous puncture to the lesion of the vertebral body after the injection of bone cement in order to increase the strength and stability of the vertebral body [7–9]. Percutaneous kyphoplasty (PKP) is a new technique developed on the basis of PVP, in which a balloon is used to create a cavity in the vertebral body before bone cement is injected [10–12]. Although PVP and PKP have significant effects in the treatment of vertebral compression fractures, there are still many complications. Therefore, it is extremely important to analyze the risk factors of postoperative complications in elderly patients with osteoporotic spinal compression fractures. The purpose of this study was to investigate the efficacy of PVP and PKP in the treatment of elderly osteoporotic spinal compression fractures and to analyze the related factors that affect the occurrence of postoperative complications. The specific report is as follows.

The article "Analysis on the Effect of Different Surgical Methods on the Treatment of Senile Osteoporotic Spinal Compression Fractures and the Influencing Factors of Complications" was retracted in 2023. Reasons: unreliable results or conclusions; concerns about the data; concerns about the peer review; concerns about the citations.

## 2. Materials and Methods

### 2.1. Patients

A total of 132 elderly patients with osteoporotic spinal compression fracture admitted to our hospital from March 2018 to December 2019 were selected as the research objects. Inclusion criteria were as follows: injury time ≤1 month; bone mineral density test *T*-value ≤ −2.5, diagnosed with osteoporosis; all of them were confirmed as spinal compression fracture by MRI, X-ray, and other imaging examinations; no pedicle damage; complete clinical data; and follow-up for nonshedding patients. Exclusion criteria were as follows: those with pathological vertebral fractures; those with hemorrhagic diseases; those with congenital immune diseases; and those with severe damage to organs, such as the liver and kidney. All patients were divided into control group and observation group with 66 cases in each group by the random number table method. In the control group, there were 38 males and 28 females, aged from 62 to 78 years, with an average age of (70.21 ± 6.14) years. In the observation group, there were 36 males and 30 females, aged 65 to 80 years, with an average age of (70.93 ± 5.69) years. There was no statistical difference between the two groups in general information (*P* > 0.05), and they were comparable. This study was approved by the ethics committee of our hospital, and informed consent was signed by the patients and their families.

### 2.2. Operation Method

All patients were placed in prone position, and cement was injected through unilateral pedicle after epidural anesthesia. The control group was treated with PVP: a percutaneous puncture along the vertebral arch was performed to locate and determine a good position. After successful puncture, the fractured vertebral body was positioned under C-arm X-ray fluoroscopy, and a 5 mm incision was made with a sharp knife at the center of the insertion point. The working cannula was replaced after the puncture was located to the appropriate position by fluoroscopy. After the working cannula was installed, the expansion tube and guide wire were removed, and the fine drill was pushed along the working cannula to the anterior edge of the vertebral body to establish the working channel. The polymethyl methacrylate (PMMA) bone cement was slowly injected into the front 1/3 of the vertebral body, and the injection was stopped after the bone cement was evenly filled in the vertebral body. After coagulation, the wound was pressed, and the incision was sutured 3∼5 min later.

The article "Analysis on the Effect of Different Surgical Methods on the Treatment of Senile Osteoporotic Spinal Compression Fractures and the Influencing Factors of Complications" was retracted in 2023. Reasons: unreliable results or conclusions; concerns about the data; concerns about the peer review; concerns about the citations.

The observation group was treated with PKP: The working channel was established by the same operation as the control group, and the balloon was inserted in the rear quarter of the vertebral body. The balloon was slowly compressed and expanded until the height of the vertebral body recovered, and then the balloon was pulled out. Under the X-ray fluoroscopy, the prepared PMMA bone cement was injected into the vertebral body.

All patients were treated with antiosteoporosis drugs after surgery, got out of bed the same day after surgery, and guided rehabilitation exercises and other postoperative treatments.

### 2.3. Observation Index

The curative effect was evaluated 2 months after the operation, and the curative effect was divided into 3 levels: “excellent” indicates most of the compressed vertebral body returns to normal state, fracture healing, no discomfort in the waist, and complete or basic recovery of function; “effective” indicates fracture healing, low back pain basically disappeared, and lumbar appearance and vertebral body shape improved compared with preoperative; and “ineffective” indicates local pain, no change in local deformity, and dysfunction. Total effective rate = (excellent + effective) number of cases/total number of cases × 100%.

Before and after treatment, the visual analogue scale (VAS) was used to evaluate the pain status of patients in both groups, with a total score of 0 to 10. The higher the score, the more severe the pain. The Oswestry Disability Index (ODI) was used to evaluate the spinal function of patients in both groups. The total score ranged from 0 to 100. The higher the score, the more severe the disability. The changes in vertebral height and the number of Cobb angles were measured by lateral radiographs before and after treatment. All patients were followed up for 6 months, and their complications were recorded.

The article "Analysis on the Effect of Different Surgical Methods on the Treatment of Senile Osteoporotic Spinal Compression Fractures and the Influencing Factors of Complications" was retracted in 2023. Reasons: unreliable results or conclusions; concerns about the data; concerns about the peer review; concerns about the citations.

### 2.4. Statistical Method

The results of this experiment were statistically analyzed by SPSS 20.0 (SPSS Co., Ltd., Chicago, USA). Count data were expressed by (rate), and chi-square test was used for their comparison between groups. Measurement data were expressed by (mean ± standard deviation), and *t*-test was used for their comparison between groups. Multivariate analysis adopts the multiple logistic regression model. *P* < 0.05 indicates that the difference is statistically significant.

## 3. Results

### 3.1. Comparison of the Efficacy of the Two Groups

In the control group, 26 cases were excellent, 32 cases were effective, and 8 cases were ineffective, with a total effective rate of 87.88%. In the observation group, 29 cases were excellent, 35 cases were effective, and 2 cases were ineffective, with a total effective rate of 96.97%. The total effective rate of observation group was higher than that of control group (*P* < 0.05), as shown in Figure 1.

### 3.2. Comparison of VAS Score and ODI Score between the Two Groups

After treatment, the VAS score and ODI score of the two groups were lower than before treatment (*P* < 0.05), as shown in Figure 2.

### 3.3. Comparison of Vertebral Body Height and Cobb Angle between the Two Groups

After treatment, the vertebral body heights of the two groups were higher than before treatment, and the Cobb angles were lower than before treatment. The vertebral body heights of the observation group were higher than those of the control group, and the Cobb angles were lower than that of the control group (*P* < 0.05), as shown in Figure 3.

### 3.4. Comparison of Complications between the Two Groups

During the follow-up period, the control group had 10 cases of bone cement leakage, 2 cases of chronic pain, and 3 cases of adjacent vertebral fractures, and the total incidence was 22.72%. In the observation group, there were 3 cases of bone cement leakage, 1 case of chronic pain, and 2 cases of adjacent vertebral fractures, and the total incidence was 9.09%. The total incidence of complications in the observation group was lower than that in the control group (*P* < 0.05), as shown in Figure 4.

### 3.5. Analysis of Univariate Factors Influencing Postoperative Complications

Univariate analysis showed that age, BMI, history of fracture, type of fracture, bone mineral density, use of hormones, and antiosteoporosis treatment were related to the occurrence of postoperative complications (*P* < 0.05), as shown in Table 1.

### 3.6. Analysis of Multiple Factors Affecting Postoperative Complications

Multivariate logistic analysis showed that age, bone mineral density, use of hormones, and antiosteoporosis treatment were independent factors affecting the occurrence of postoperative complications (*P* < 0.05), as shown in Tables 2 and 3.

The article "Analysis on the Effect of Different Surgical Methods on the Treatment of Senile Osteoporotic Spinal Compression Fractures and the Influencing Factors of Complications" was retracted in 2023. Reasons: unreliable results or conclusions; concerns about the data; concerns about the peer review; concerns about the citations.

## 4. Discussion

Osteoporosis is a metabolic disease that often occurs in the elderly. Patients with decreased bone mass, bone tissue degradation, and high bone fragility are often associated with the risk of fracture [13, 14]. Among them, spinal compression fracture is relatively common. After fracture, patients have limited mobility and often accompanied by spinal pain, which requires timely and effective treatment. Otherwise, complications such as delayed fracture healing and bone nonunion will occur, which will seriously affect the quality of life of patients [15–17]. The common treatment methods are conservative treatment and surgical treatment. Conservative treatment includes bed rest, medication analgesia, rehabilitation treatment, and bracing. Although pain symptoms can be relieved after conservative treatment, however, due to the limited activities in bed for a long time can lead to osteoporosis increase, lower extremity deep vein thrombosis, pulmonary infection, urinary tract infection and stone and bedsore complications, such as serious influence quality of life, and disability fatality rate is high, can bring serious damage to family and social burden of economy and society. In addition, in the later stage of conservative treatment, vertebral height loss, local kyphosis, recurrent fracture, chronic low back pain, and other sequelae may occur [18, 19]. Traditional surgery mainly uses the pedicle screw technique for treatment. Due to the loss of vertebral bone mass, sparse bone trabeculae, vertebral compressive strength, and significant decrease of pedicle screw holding, it is easy to cause postoperative pedicle screw loosening, failure, and vertebral recollapse. Currently, PVP and PKP are the main clinical surgical treatments, both of which are minimally invasive surgery with short operation time, effective pain relief, and rapid postoperative recovery. The main difference between the two is that PKP uses a balloon to complete the reduction of the vertebral body with the help of balloon expansion [20–22]. Although both can achieve good curative effects, there is still controversy about the pros and cons of the two in the treatment of osteoporotic spinal compression fractures. Our hospital has a wealth of clinical experience in the treatment of spinal compression fractures. This study summarizes our physicians' years of experience in the treatment of spinal compression fractures to provide a certain reference for clinical applications.

The article "Analysis on the Effect of Different Surgical Methods on the Treatment of Senile Osteoporotic Spinal Compression Fractures and the Influencing Factors of Complications" was retracted in 2023. Reasons: unreliable results or conclusions; concerns about the data; concerns about the peer review; concerns about the citations.

The results of this study showed that after treatment, the VAS scores and ODI scores of the two groups were lower than those before treatment. It shows that both surgical methods can effectively improve the patient's pain and dysfunction. The reason is that PVP and PKP eliminate micro fractures caused by fretting through the fixation of bone cement and stabilize the stability of the spine. On the other hand, the heat released during the solidification of bone cement damages the nerve endings of pain sensation and blocks the conduction of pain sensation. Moreover, the monomer toxic effect of bone cement can also injure the pain-sensitive nerve endings, relieve pain, and effectively relieve the pressure in the vertebral body, increasing the strength of bone and the stability of the vertebral body, so as to effectively maintain the normal function of patients [23–26]. The results of this study showed that the total effective rate of the observation group was higher than that of the control group. After treatment, the vertebral bodies' height in the two groups was higher than before treatment, and the Cobb angle was lower than before treatment, and the vertebral body height in the observation group was higher than that of the control group, and the Cobb angle was lower than that of the control group. These results indicated that both groups could effectively recover vertebral height and correct kyphosis, but PKP was better than PVP. The reason is that the high-pressure injection of PVP and the fluidity of the bone cement make it easy for the bone cement to leak into the vertebrae and damage the spinal cord and nerve roots, which reduces the effect of the operation to a certain extent. PKP is an improved procedure based on PVP. The vertebral body is fully expanded by a balloon to form a closed osseous cavity in the vertebral body, and then bone cement is injected into the balloon to restore the vertebral height by compaction and expansion of the vertebral body [27, 28]. Therefore, PKP can significantly reduce the risk of bone cement leakage and significantly improve the deformed spine.

The chemical composition and curing reaction of different bone cements are different, which may cause allergic reaction, monomer toxicity, and local foreign body reaction after injection into the body. If bone cement particles enter the blood circulation, there is a risk of tissue and organ embolism, especially pulmonary embolism [29, 30]. For the cement to be successfully injected into the vertebral body, a certain amount of injection pressure and fluidity (viscosity) is required, which allows the cement to leak out of the vertebral body through the venous plexus of return, fracture, or bone defect, squeezing or burning surrounding tissues [31, 32]. The vast majority of cement leakage does not cause significant clinical symptoms, but in rare cases it can result in nerve root or spinal cord injury and pulmonary embolism. The results of this study showed that during the follow-up period, 10 cases of bone cement leakage, 2 cases of chronic pain, and 3 cases of adjacent vertebral body fracture and other complications occurred in the control group, with a total incidence of 22.72%. In the observation group, there were 3 cases of bone cement leakage, 1 case of chronic pain, and 2 cases of adjacent vertebral body fracture and other complications, with a total incidence of 9.09%. The total incidence of complications in the observation group was lower than that in the control group. It shows that the safety of PKP is higher than that of PVP. Our doctors learn and discuss with each other through surgical operations, postoperatively, and summarize their experiences as follows. Due to the need for prone position during the operation and most of the patients are elderly with poor physical strength, appropriate tolerance training can be carried out before the operation. Bone cement injection may cause cardiovascular system reaction in patients. Therefore, blood pressure, heart rate, and other vital signs should be closely observed during the operation. After surgery, the patients were observed for dyspnea, cough, chest tightness, numbness in lower limbs, and other symptoms to avoid bone cement leakage. The risk of bone cement leakage can be reduced by correctly grasping the injection timing, injection volume, and injection method.

The article "Analysis on the Effect of Different Surgical Methods on the Treatment of Senile Osteoporotic Spinal Compression Fractures and the Influencing Factors of Complications" was retracted in 2023. Reasons: unreliable results or conclusions; concerns about the data; concerns about the peer review; concerns about the citations.

In this study, multivariate logistic analysis showed that age, bone mineral density, use of hormones, and antiosteoporosis treatment were independent factors influencing the occurrence of postoperative complications. The reason is that as the patient ages, the more serious the loss of calcium in the body, the more porous the bone, and the worse the body function and recovery function, which affects the patient's postoperative recovery. Patients with low bone density have relatively loose bones and higher bone fragility, which greatly increases the probability of adjacent vertebral body fractures [33, 34]. The use of hormones can inhibit the survival of bone cells, further aggravate the degree of osteoporosis, and increase the risk of refracture after surgery [35, 36]. Antiosteoporosis therapy can effectively reduce bone resorption, improve the bone quality of patients, and improve their weight-bearing status. Therefore, postoperative antiosteoporosis therapy can effectively avoid the occurrence of fractures, thus improving the prognosis of patients [37, 38].

The article "Analysis on the Effect of Different Surgical Methods on the Treatment of Senile Osteoporotic Spinal Compression Fractures and the Influencing Factors of Complications" was retracted in 2023. Reasons: unreliable results or conclusions; concerns about the data; concerns about the peer review; concerns about the citations.

## 5. Conclusion

In summary, both PVP and PKP can effectively improve the pain and dysfunction of elderly patients with osteoporotic spinal compression fracture, restore vertebral height, and correct kyphosis, but PKP has better effect and higher safety and is worth promoting. Postoperative complications of patients are related to their age, bone mineral density, use of hormones, and antiosteoporosis treatment.

## Figures and Tables

**Figure 1:** Comparison of the efficacy of the two groups. *Note*. Compared with the control group, ^*∗*^*P* < 0.05.

**Figure 2:** Comparison of (a) VAS score and (b) ODI score between the two groups. *Note*. Compared with before treatment, ^*∗*^*P* < 0.05.

**Figure 3:** Comparison of (a) vertebral body height and (b) Cobb angle between the two groups. *Note*. Compared with before treatment, ^*∗*^*P* < 0.05. Compared with the control group, ^#^*P* < 0.05.

**Figure 4:** Comparison of complications between the two groups. *Note*. Compared with the control group, ^*∗*^*P* < 0.05.

**Table 1:** Analysis of univariate factors influencing postoperative complications.

Factors	*n*	The normal group (*n* = 111)	The complication group (*n* = 21)	*χ* ^*2*^	*P*
Age (year)				3.889	0.048
≤70	70	63 (56.76%)	7 (33.33%)		
>70	62	48 (43.24%)	14 (66.67%)		

Sex				1.141	0.285
Male	74	60 (54.05%)	14 (66.67%)		
Female	58	51 (45.95%)	7 (33.33%)		

BMI (kg/m^2^)				5.301	0.021
≤19	52	39 (35.14%)	13 (61.90%)		
>19	80	72 (64.86%)	8 (38.10%)		

Hypertension				0.655	0.418
Yes	48	42 (37.84%)	6 (28.57%)		
No	84	69 (62.16%)	15 (71.43%)		

Diabetes				0.462	0.497
Yes	26	23 (20.72%))	3 (14.29%)		
No	106	88 (79.28%)	18 (85.71%)		

History of fracture				5.467	0.019
Yes	46	34 (30.63%)	12 (57.14%)		
No	86	77 (69.37%)	9 (42.86%)		

Type of fracture				5.726	0.017
Wedge	69	53 (47.75%)	16 (76.19%)		
Nonwedge	63	58 (52.25%)	5 (23.81%)		

Bone mineral density (SD)				4.659	0.031
1.0∼2.5	48	36 (32.43%)	12 (57.14%)		
>2.5	84	75 (67.57%)	9 (42.86%)		

Use of hormones				6.241	0.012
Yes	34	24 (21.62%)	10 (47.62%)		
No	98	87 (78.38%)	11 (52.38%)		

Antiosteoporosis treatment				5.344	0.021
Yes	106	93 (83.78%)	13 (61.90%)		
No	26	18 (16.22%)	8 (38.10%)		

**Table 2:** Assignment for multivariate analysis of factors.

Factors	Variable	Assignment
Age	X1	≤70 = 0, >70 = 1
BMI	X2	>19 = 0, ≤19 = 1
History of fracture	X3	No = 0, yes = 1
Type of fracture	X4	Non-wedge = 0, wedge = 1
Bone mineral density	X5	>2.5 = 0, 1.0∼2.5 = 1
Use of hormones	X6	Yes = 0, no = 1
Antiosteoporosis treatment	X7	Yes = 0, no = 1

**Table 3:** Analysis of multiple factors affecting postoperative complications.

Variables	*B*	SE	Walds	*P*	OR	95% CI
Age	1.185	0.432	4.416	0.038	3.271	1.694∼6.815
BMI	0.402	0.184	1.936	0.215	1.494	0.782∼2.139
History of fracture	0.485	0.212	1.896	0.281	1.624	0.904∼2.216
Type of fracture	0.368	0.176	1.369	0.354	1.445	0.859∼2.024
Bone mineral density	1.289	0.506	5.015	0.026	3.629	1.982∼5.839
Use of hormones	1.324	0.681	5.698	0.019	3.758	1.269∼7.306
Antiosteoporosis treatment	1.175	0.483	5.265	0.023	3.238	1.756∼4.892

The article "Analysis on the Effect of Different Surgical Methods on the Treatment of Senile Osteoporotic Spinal Compression Fractures and the Influencing Factors of Complications" was retracted in 2023. Reasons: unreliable results or conclusions; concerns about the data; concerns about the peer review; concerns about the citations.

## Data Availability

The data can be obtained from the corresponding author upon reasonable request.
